RETRACTED

# Analysis of the Effect of Rational Emotional Intervention Combined with Hierarchical Management Mode on Improving the Psychological Stress of Emergency Nurses and Trainee Nurses

**DOI:** 10.1155/2022/2038018

**Published:** 2022-06-10

**Authors:** Shirui Liu, Xiangsu Li, Xianghong Yin, Liqun Wang

**Affiliations:** ^1^College of Educational Science, Hengyang Normal University, Hengyang 421002, Hunan, China; ^2^Health School of Nuclear Industry, Hengyang 421002, Hunan, China; ^3^The Affiliated Nanhua Hospital, Hengyang Medical School, University of South China, Hengyang 421002, Hunan, China

## Abstract

**Purpose:**

To explore the effect of rational emotional intervention combined with hierarchical management mode on improving the psychological stress of emergency nurses and trainee nurses.

**Methods:**

50 emergency nurses who worked or practiced in our hospital from June 2019 to May 2021 were selected as the research object. From June 2019 to May 2020, our hospital adopted the traditional management mode. From June 2020 to May 2021, our hospital adopted the rational emotional intervention combined with hierarchical management mode. The psychological state, work stress, stress response, job burnout, and sleep quality of emergency nurses were compared before and after intervention.

**Results:**

Compared with before intervention, the scores of self-rating anxiety scale and self-rating depression scale, the work stress scores, the Maslach burnout inventory score, the Pittsburgh sleep quality index score of emergency nurses decreased after intervention (*P* < 0.05). Compared with before intervention, the stress coping scores of emergency nurses increased after intervention (*P* < 0.05).

**Conclusion:**

The rational emotional intervention combined with hierarchical management mode can improve the psychological pressure of emergency nurses and trainee nurses, reduce job burnout, improve stress coping ability, and improve sleep quality.

## 1. Introduction

The emergency department is the department for receiving patients with acute and critical diseases and sudden diseases. Most of the patients have serious diseases, rapid development, many emergencies, short rescue time, and large patient turnover [1]. Therefore, emergency nurses are overloaded with work for a long time, with great mental pressure, serious job burnout, and poor sleep quality, thus affecting the quality of nursing. For trainee nurses, it can lead to lower job expectancy [2]. When the nursing work is not divided according to the nurses' personal ability and the nurse feels unable to be competent for the job, the nurses often have anxiety and depression, and work in a negative state, and the physiological and psychological pressure cannot be effectively regulated, resulting in the increase of the probability of nursing error events [3]. At the same time, emergency department trainee nurses are the backup force of clinical nursing services. After trainee nurses entering clinical practice, the external environment, interpersonal relationships, and learning methods will change, coupled with the pressure brought by the nursing profession itself, which will have a certain impact on the study, physiological and psychological activities of trainee nurses. Therefore, how to reduce the work pressure or study pressure of emergency nurses and trainee nurses is one of the key topics studied of nursing management. Rational emotional intervention is an intervention method that replaces irrational thinking mode with rational thinking mode. Its core value is rational manipulation of irrationality so as to help people change their bad cognition and reduce or even eliminate negative emotions caused by induced events [4, 5]. Hierarchical management mode is to accurately identify the development level of the management object, and then design the corresponding level management method by identifying the development level of the object. This method can realize effective management at all levels and improve nurses' enthusiasm for nursing work through reasonable arrangement of their work and responsibilities [6, 7]. The purpose of this study is to observe the application effect of rational emotional intervention combined with hierarchical management mode in emergency nurses and trainee nurses.

RETRACTED

## 2. Materials and Methods

### 2.1. Research Object

50 emergency nurses who worked or practiced in our hospital from June 2019 to May 2021 were selected as the research object. Among them, there were 46 females and 4 males. The average age was (25.75±2.64) years. Education level: 10 cases were secondary vocational nursing students, 3 cases were junior college nursing students, 5 cases were undergraduate nursing students, 9 cases were junior college, 22 cases were undergraduate, and 1 case was master. Professional title: 13 cases were trainee nurses, 25 cases were nurses, 5 cases were nurse practitioner, 4 cases were nurse-in-charge, 2 cases were cochief superintendent nurse, and 1 case was chief superintendent nurse. Inclusion criteria: emergency nurses who worked in the emergency department of our hospital and have been engaged in emergency nursing >1 year. During the study period, the emergency nurses who worked in our hospital for internship, advanced study, or rotation. Volunteer to participate in this research. Exclusion criteria: nurses who have been absent or absent for a long time during the study period; trainee nurses who were transferred to other departments during the study period; nurses with a history of mental illness; nurses who have experienced severe stress reactions before this study; nurses with severe organic diseases themselves.

RETRACTED

### 2.2. Research Methods

From June 2019 to May 2020, our hospital adopted the traditional management mode. Emergency nurses regularly receive theoretical knowledge, carry out practical skills training, and implement routine management methods such as reward and punishment management and system management. Trainee nurses were taught by a senior teacher under the “one-to-one” teaching model. In addition, emergency nurses needed to give psychological lectures, emotional counseling, and other routine psychological care.

From June 2020 to May 2021, our hospital adopted the rational emotional intervention combined with hierarchical management mode.

- Rational emotional intervention: once a week, each time for 1 h. Psychological diagnosis stage: in a quiet environment, fully communicate with emergency nurses to understand the reasons for their nervousness, anxiety, and stress. To observe the emotional manifestations of emergency nurses and find out the reasons for their poor psychological state. It was especially necessary to pay attention to the psychological pressure of trainee nurses, communicate with trainee nurses regularly, understand the problems existing in the practice, and provide clinical guidance to trainee nurses in a targeted manner. Comprehension stage: the corresponding events were analyzed according to the known reasons, and representative emotional events were collected. Point out the reasonable and unreasonable place of the nurse when facing the event, and guide the nurse to be aware of these unreasonable thoughts in time. Emergency department nurses were instructed to control their own pressure, to eliminate absolutism and excessive disaster thinking, and to change the nurses' own thinking. When emergency department nurses faced with the failure of rescue events, nurses should control their mentality, avoid panic, self-blame, and other emotions. Make nurses realize that inducing events will not directly lead to bad psychology and stress but subjective consciousness. Only by changing irrational beliefs can we alleviate the existing symptoms. For trainee nurses, it is necessary to carry out the training of positive response to pressure regularly so that trainee nurses can correctly understand and deal with setbacks, and timely through the correct way to relieve negative emotions. Revision stage: emergency nurses were encouraged to debate their irrational beliefs and explore emotions and thoughts that were inconsistent with positive results. Emergency nurses were instructed to establish reasonable beliefs and face adverse events from a positive perspective so as to change their own emotions and behaviors. Reeducation stage: consolidate the effect of the previous stage of treatment and help emergency nurses to re-establish new coping styles in cognitive style, thinking process, emotional and behavioral performance, etc. Instruct emergency nurses to use what they have learned to deal with problems in their future work and life. At the same time, instruct trainee nurses to correctly understand the difference between work problems and textbook knowledge, and make up for the lack of textbooks in the emotional management of emergency department work.
- Hierarchical management mode: the level of each layer was set up according to the factors such as nurses' working time, professional level, professional title, and education level in the emergency department, the research objects are divided into head nurses, senior responsible nurses, junior responsible nurses, auxiliary nurses, and trainee nurses. Evaluate the emergency nurses in many aspects, arrange their work according to their individual personalities and specialties, and optimize the combination of nurses. For nurses with bad psychological pressure, decompression should be given and division of labor should be adjusted. Hierarchical training: pay attention to strengthening the training of basic knowledge and professional skills. The training object is mainly auxiliary nurses and trainee nurses, the training content is related nursing knowledge of emergency nursing, and the main responsible persons are head nurses and responsible nurses; train organizational ability and conduct hierarchical training. The head nurse is responsible for training the responsible nurse, and the responsible nurse is responsible for training the assistant nurse. Hierarchical management: the work content of grade 1–5 emergency nurses was reasonably arranged according to the actual situation. In the past, problems existing in nursing operation of nurses of different levels were found in time, and problems were reported layer by layer, and then the problems were dealt with. Trainee nurses carry out hierarchical and staged practice, and independently complete different stages of work under the guidance of nurses at all levels. See Table 1 for the specific responsibilities of nurses at all levels.

RETRACTED

### 2.3. Observation Index

All questionnaires were conducted by secret ballot. Before and after the intervention, 50 questionnaires were distributed and 50 questionnaires were collected, with an effective recovery rate of 100%.

- Self-rating anxiety scale (SAS) and self-rating depression scale (SDS) were used to evaluate psychological state. There were 20 items in SAS, and the 4-level scoring method was adopted, with the demarcation value of 50 points. There were 20 items in SDS, with a 4-level scoring method was adopted, with the demarcation value of 53 points. The higher the score, the worse the psychological state. The Cronbach's *α* coefficient of SAS was 0.834. The Cronbach's *α* coefficient of SDS was 0.819.
- The nurses' work stress scale was used to evaluate the work stress including 5 dimensions, nursing profession and work, time allocation and workload, working environment and equipment, patient nursing, management, and interpersonal. The 4-level scoring method was adopted. The higher the score, the greater the pressure in this dimension. The Cronbach's *α* coefficient of the scale was 0.757.
- The coping style questionnaire was used to evaluate the stress coping situation including 6 dimensions, solve the problem, self-blame, ask for help, fantasize, retreat, and rationalize. The higher the score, the better the coping style of this dimension. The Cronbach's *α* coefficient of the questionnaire was 0.720.
- Maslach Burnout Inventory (MBI) was used to evaluate job burnout including 22 items, with a total score of 132 points by using the 7-level scoring method. The higher the score, the stronger the job burnout. The Cronbach's *α* coefficient of MBI was 0.783.
- Pittsburgh Sleep Quality Index (PSQI) was used to evaluate sleep quality including 19 self-evaluation items and 5 other evaluation items, with a total score of 21 points by using the 4-level scoring method. The higher the score, the worse the sleep quality. The Cronbach's *α* coefficient of PSQI was 0.806.

### 2.4. Statistical Methods

The SPSS 22.0 software (Armonk, NY; IBM Corp) was used for analysis. The measurement data were expressed as mean ± standard deviation, and *t*-test was used to analyze the comparison. *P* < 0.05 was statistically significant.

## 3. Results

### 3.1. Comparison of Psychological State before and after Intervention

Compared with before intervention, the scores of SAS and SDS of emergency nurses decreased after intervention (*P* < 0.05), as shown in Figure 1.

Compared with before intervention, the work stress scores of emergency nurses decreased after intervention (*P* < 0.05) as shown in Figure 2.

Compared with before intervention, the stress coping scores of emergency nurses increased after intervention (*P* < 0.05) as shown in Figure 3.

Compared with before intervention, the MBI score of emergency nurses decreased after intervention (*P* < 0.05) as shown in Figure 4.

RETRACTED

Compared with before intervention, the PSQI score of emergency nurses decreased after intervention (*P* < 0.05) as shown in Figure 5.

## 4. Discussion

The emergency department has many emergencies accidents and complicated work. Compared with other departments, the nurse-patient relationship is more tense, and medical disputes are more likely to occur. In the heavy and tense working environment, emergency nurses suffer from great psychological pressure, which comes from high work intensity, no guidance to solve problems, poor professional identity, and so on. In particular, the trainee nurses who have just entered the hospital environment are relatively young, and most of them are not strong in self-psychological regulation, and have insufficient understanding of nursing practice, which will affect the mental health of the trainee nurses [8, 9]. In the traditional nursing management, the responsibilities and obligations of nursing posts is not clear, the nursing management efficiency is low, the psychological feelings of nurses are ignored, and the division of labor among nurses is only based on the professional level and professional title of nurses. It is easy to cause the negative emotions of emergency nurses, seriously affecting the sleep quality of nurses, and then affecting the clinical outcome of patients [10].

Reasonable emotional intervention method believes that inducing events will not directly lead to bad psychology and stress, but subjective consciousness. Only by changing irrational beliefs can people relieve and remove their emotional troubles and form positive behavioral responses and emotional changes [11, 12]. Ghawadra et al. showed that reasonable emotional intervention measures can improve people's cognition of events, abandon previous unreasonable ideas, establish a new mode of thinking, and guide them to consider the occurrence and development of events with reasonable thinking, which is conducive to promoting people's mental health [13]. Based on scientific management and behavior management, hierarchical management mode implements hierarchical responsibility system, which can rationally allocate human resources and reduce unnecessary waste of nursing resources [14, 15]. Kawaguchi et al. believed that through hierarchical management, clarifying the job responsibilities of nurses at all levels, and through measures such as layer by layer supervision and guidance, it can give staff at all levels of work autonomy and enthusiasm, and reduce the pressure at work [16].

In this study, the application of rational emotional intervention combined with hierarchical management mode can reduce SAS, SDS, job stress, MBI, and PSQI scores of emergency nurses, and improve their stress coping scores. We believe that the results show that this intervention program can improve the psychological stress of emergency nurses and trainee nurses, reduce job burnout, improve stress coping ability, and improve sleep quality. The reason may be rational emotional intervention guides emergency nurses through 4 stages of psychological diagnosis, comprehension, revision, and reeducation, find out the specific reasons for their poor psychological state, positively guide their thinking consciousness, and help emergency nurses reshape the correct way of thinking [17]. Also, it can change nurses' cognition of adverse events so that they can face the pressure correctly. This method encourages emergency nurses to debate with their irrational beliefs, adopt positive coping styles to eliminate absolute views and ideas, and take practical actions to control their emotions reasonably so as to finally reduce the harm caused by psychological stress and improve their sleep level [18, 19]. In addition, after the hierarchical management of emergency nurses, we carry out targeted training according to different levels of nurses so that the human resources can be optimally allocated and the nursing quality can be improved [20]. Reasonable distribution of nursing responsibilities can promote the mutual help of nurses at different levels in the group and can reduce the intensity of nursing work, which has a positive effect on reducing the psychological pressure of emergency nurses and improving the quality of sleep [21]. Through the step-by-step supervision of the emergency department, the superior nurses can effectively understand the working level of the junior nurses, timely find and guide the problems and mistakes encountered in the nursing operation, eliminate the doubts of the nurses in the work, is conducive to reduce the pressure of the junior nurses due to the lack of emergency nursing ability, and enhance the ability to cope with pressure [22]. In the implementation of the hierarchical management mode, junior nurses can play an assisting role in the rescue work so that senior nurses can keep their mental focus during the rescue [23]. At the same time, this model can prevent senior nurses from engaging in simple work, make nurses at all levels undertake different nursing tasks, and promote emergency nurses to concentrate on nursing work, thus effectively reduce the job burnout of nurses [24]. We combine rational emotional intervention with hierarchical management mode in emergency nurses, which can learn from each other's strengths and complement each other's weaknesses. The two intervention methods play a synergistic role, resulting in a more significant improvement of the psychological stress of emergency nurses and trainee nurses.

RETRACTED

It is worth noting that for trainee nurses, traditional management methods can only train nurses at a single level, and tend to ignore the psychological pressure of nurses, and lack all-round practice teaching. Rational emotional intervention can enable trainee nurses to study and work in a healthy physical and mental state under moderate stress, and enhance trainee nurses' sense of professional achievement through regular training on occupational stress management and active response to stress. At the same time, this method can help interns in clinical practice as soon as possible to eliminate tension and anxiety so that the trainee nurses can keep a positive attitude and look at the nursing work with a happy mood. After implementing hierarchical practice for trainee nurses, by adjusting the work intensity from light to heavy according to the nurse's ability, the nursing ability can be cultivated step by step, and the enthusiasm of the nurses to work can be improved comprehensively, and the work pressure can be reduced. The hierarchical management mode can fully explore the potential of trainee nurses, reduce the job burnout of trainee nurses, enhance career aspirations, so as to lay a solid foundation for becoming a qualified nurse in the future.

## 5. Conclusion

To sum up, rational emotional intervention combined with hierarchical management mode can improve the psychological pressure of emergency nurses and trainee nurses, reduce job burnout, improve stress coping ability, and improve sleep quality. The research time of this study is short, and it remains to be further observed the long-term application effect of rational emotional intervention combined with hierarchical management mode in emergency nurses.

## Figures and Tables

**Figure 1:** Comparison of psychological state before and after intervention compared with before intervention, ^*∗*^*P* < 0.05. Comparison of work stress before and after intervention.

**Figure 2:** Comparison of work stress before and after intervention compared with before intervention, ^*∗*^*P* < 0.05. Comparison of stress response before and after intervention.

**Figure 3:** Comparison of stress response before and after intervention compared with before intervention, ^*∗*^*P* < 0.05. Comparison of job burnout before and after intervention.

**Figure 4:** Comparison of job burnout before and after intervention compared with before intervention, ^*∗*^*P* < 0.05. Comparison of sleep quality before and after intervention.

**Figure 5:** Comparison of sleep quality before and after intervention compared with before intervention, ^*∗*^*P* < 0.05.

RETRACTED

**Table 1:** Specific responsibilities of nurses at all levels.

Hierarchy	Professional title	Levels	Specific work content
Trainee nurses	Nursing students	Level 1	Early-practice: under the guidance of level 2 nurses, the students will initially master the nursing procedures, strengthen the basic nursing operations, and apply them to practical nursing, so as to meet the patients' basic life nursing Mid-practice: under the guidance of level 3 nurses, the students will be able to independently complete the work of an assistant nurse, master common nursing skills, and strengthen the skills of specialist operation, disease observation, writing nursing records, handover, and nurse-patient communication and so on Late-practice: under the guidance of level 4 nurses, the students will be able to skillfully apply nursing procedures, strengthen comprehensive nursing level, and continuously improve the overall ability of nursing work and the ability to complete it independently

Auxiliary nurses	Nurse	Level 2	Under the guidance of level 3 nurses, be responsible for assisting the responsible nurses to implement basic specialist care and life care for patients; observe the patient's vital signs and report any abnormal situation to the doctor in time; participate in the formulation of nursing plan, implement targeted nursing for patients, and strengthen communication with patients

Junior responsible nurses	Nurse practitioner and above	Level 3	Under the guidance of level 4 nurses, responsible for the clinical nursing and treatment of patients from admission to discharge; check the patient's medical records, and assist doctors in ward management; responsible for the teaching work of some level 1 nurses; carry out health education and discharge guidance for patients and their families

Senior responsible nurses	Nurse-in-charge and above	Level 4	Under the guidance of level 5 nurses, organize ward rounds and training of junior nurses; responsible for communication and coordination, organizing and completing the rescue work for patients; organize the training of nurses in emergency department, and adjust the psychological pressure of nurses

Head nurses	Cochief superintendent nurse, chief superintendent nurse	Level 5	Responsible for overall scheduling and supervision, guiding the work of junior nurses, and solving the problems existing in junior nurses; manage resources and prepare rescue items; research new nursing technology, participate in nursing academic conferences, etc

## Data Availability

The data used and/or analyzed during the current study are available from the corresponding author.
